The article "Blood Flow and Shear Stress Allow Monitoring of Progression and Prognosis of Tumor Diseases" was published in 2021. Journal: Front Physiol.

# Blood Flow and Shear Stress Allow Monitoring of Progression and Prognosis of Tumor Diseases

**DOI:** 10.3389/fphys.2021.693052

**Published:** 2021-08-03

**Authors:** Matthias Barral, Imane El-Sanharawi, Anthony Dohan, Maxime Sebuhyan, Alexis Guedon, Audrey Delarue, Alexandre Boutigny, Nassim Mohamedi, Benjamin Magnan, Salim Kemel, Chahinez Ketfi, Nathalie Kubis, Annouk Bisdorff-Bresson, Marc Pocard, Philippe Bonnin

**Affiliations:** ^1^INSERM UMR1275, Université de Paris, Hôpital Lariboisière, Paris, France; ^2^AP-HP, Université de Paris, Hôpital Lariboisière, Physiologie Clinique – Explorations Fonctionnelles, Paris, France; ^3^INSERM UMR1148 - LVTS, Université de Paris, Hôpital Bichat, Paris, France; ^4^AP-HP, Université de Paris, Hôpital Lariboisière, Neuroradiologie, Centre Constitutif des Malformations Artério Veineuses Superficielles de l'Enfant et de l'Adulte, Paris, France; ^5^AP-HP, Sorbonne-Université, Hôpital Pitié-Salpêtrière, Chirurgie Digestive et Cancérologique, Paris, France

**Keywords:** wall shear stress, blood flow velocity, superior mesenteric artery, peritoneal carcinomatosis, pseudomyxoma peritonei, carotid artery, arteriovenous malformation, disease progression

## Abstract

In the presence of tumor angiogenesis, blood flow must increase, leading to an elevation of blood flow velocities (BFVels) and wall shear stress (WSS) in upstream native arteries. An adaptive arterial remodeling is stimulated, whose purpose lies in the enlargement of the arterial inner diameter, aiming for normalization of BFVels and WSS. Remodeling engages delayed processes that are efficient only several weeks/months after initiation, independent from those governing expansion of the neovascular network. Therefore, during tumor expansion, there is a time interval during which elevation of BFVels and WSS could reflect disease progression. Conversely, during the period of stability, BFVels and WSS drop back to normal values due to the achievement of remodeling processes. Ovarian peritoneal carcinomatosis (OPC), pseudomyxoma peritonei (PMP), and superficial arteriovenous malformations (AVMs) are diseases characterized by the development of abnormal vascular networks developed on native ones. In OPC and PMP, preoperative blood flow in the superior mesenteric artery (SMA) correlated with the per-operative peritoneal carcinomatosis index (OPC: *n* = 21, *R* = 0.79, *p* < 0.0001, PMP: *n* = 66, *R* = 0.63, *p* < 0.0001). Moreover, 1 year after surgery, WSS in the SMA helped in distinguishing patients with PMP from those without disease progression [ROC-curve analysis, AUC = 0.978 (0.902–0.999), *p* < 0.0001, sensitivity: 100.0%, specificity: 93.5%, cutoff: 12.1 dynes/cm^2^]. Similarly, WSS in the ipsilateral afferent arteries close to the lesion distinguished stable from progressive AVM [ROC-curve analysis, AUC: 0.988, (0.919–1.000), *p* < 0.0001, sensitivity: 93.5%, specificity: 95.7%; cutoff: 26.5 dynes/cm^2^]. Blood flow volume is indicative of the tumor burden in OPC and PMP, and WSS represents an early sensitive and specific vascular marker of disease progression in PMP and AVM.

The article "Blood Flow and Shear Stress Allow Monitoring of Progression and Prognosis of Tumor Diseases" was published in 2021. Journal: Front Physiol.

## Introduction

Significant physiological or pathophysiological variations of blood flow and arterial pressure occur continuously during life. For instance, an increase in metabolic demand in response to various conditions results in a transient increase of the blood flow volume (BFVol) to cover the metabolic needs. This increase is accompanied by an increase in blood flow velocity (BFVel) and wall shear stress (WSS), which stimulate endothelium-derived nitric oxide (NO) dilation (flow-mediated dilation) amounting to a 5–8% increase in the artery inner diameter (Furchgott and Zawadzki, 1980). This prompt adaptation tends to reestablish the BFVel and the WSS to resting values. Permanent exposure to increased BFVels and WSS likely leads to a continuous upregulation of the endothelial NO synthases responsible for a long-term structural arterial vascular remodeling with cellular (vascular smooth muscle cell and endothelial cell) and intercellular matrix component modifications (Rudic et al., 1998; Tronc et al., 2000). This arterial remodeling then results in arterial diameter enlargement, medial arterial wall thickening, hypertrophy, and fibrosis (Kamiya and Togawa, 1980; Davies, 1995; Tronc et al., 1996; Ben Driss et al., 1997). It has been demonstrated even in atherosclerosis and hypertension that arterial remodeling evolves over a few weeks in animal models to a few months in human (Kubis et al., 2001; Lehoux et al., 2006).

Cancer represents a pathophysiological condition in which a neoformed vascular network develops directly on the native vascular network of an organ. The neoformed vascular network is of poor quality and consists of incomplete vascular wall architecture, with direct arteriovenous fistulae and without pericytes and vascular innervation. Development of the neoformed vascular network on the native ones leads to a drop in hemodynamic resistance and a simultaneous increase in BFVol, BFVels, and WSS in the upstream native afferent conduit arteries that could consecutively initiate arterial remodeling, particularly during the periods of disease progression. The complete achievement of these processes is delayed compared to the expansion of the neoformed vascular network. The consecutive time delay (weeks, months) results in an imbalance between the arterial inflow (BFVol, BFVel, and WSS increase) and the downstream vascular network. Conversely, during periods of disease stability, the completion of the arterial remodeling leads to the normalization of the BFVel and WSS (Figures 1A–C). Of note, an expansive arterial remodeling process in carotids has been previously shown in experimental models of carotid-jugular anastomoses (Lehoux and Lévy, 2006).

The article "Blood Flow and Shear Stress Allow Monitoring of Progression and Prognosis of Tumor Diseases" was published in 2021. Journal: Front Physiol.

**Figure 1:** Schematic representation of hemodynamic modifications in the presence of an abnormal vascular network. **(A)** Normal microvascular network (μvasc.network) is interposed between the afferent native artery and the vein of drainage responsible for the hemodynamic resistance (hR) proportional to the arteriolar tone and to the microvascular density. In the upstream afferent artery, the inner diameter is adapted to maintain the blood flow velocities (BFVel), the blood flow volume (BFVol), and the wall shear stress (WSS) in normal ranges. **(B,C)** In the presence of an abnormal neoformed vascular network, the hemodynamic resistance falls due to the augmentation of the microvascular density and BFVol increases. **(B)** In the presence of a progression disease, the continuously growing downstream vascular network imposes an increase in BFVels and WSS in the afferent artery. **(C)** In the presence of a stable disease, the enlargement of the afferent artery allows to reach the balance between arterial inflow and the downstream vascular network with normalization of the BFVels and the WSS whenever the BFVol remains elevated. This normalization can therefore be recognized and reported to the stability of the vascular lesion.

Several experimental studies were initially performed to test the hypothesis of blood flow increase during tumor angiogenesis (Bonnin et al., 2007, Dohan et al., 2014). With the proof of concept established, the measurement of blood flows was therefore translated to clinical practice in patients with pseudomyxoma peritonei (PMP) (Dohan et al., 2017). Patients with face, neck, and forehead arteriovenous malformation (AVM) with high blood flows were also explored as a disease model with potential arterial remodeling (El Sanharawi et al., 2020). Fortunately in human, the BFVels and the inner diameters of the afferent arteries were measurable with enough accuracy allowing the calculation of the BFVols and WSS. Remarkably, it has recently been demonstrated in PMP and AVM that evaluating the stage of arterial remodeling could indicate disease progression thanks to only a one-time ultrasound examination performed in the afferent arteries (Barral et al., 2019; El Sanharawi et al., 2020). The present study includes a larger number of patients with ovarian peritoneal carcinomatosis (OPC), PMP, and AVM and permits to better refine the thresholds and cutoffs of BFVels, BFVols, and WSSs that help to evaluate the tumor burden and disease progression.

The article "Blood Flow and Shear Stress Allow Monitoring of Progression and Prognosis of Tumor Diseases" was published in 2021. Journal: Front Physiol.

## Clinical Relevance of the Studied Diseases

### Ovarian Peritoneal Carcinomatosis

Ovarian cancer is the most lethal gynecological malignancy, with an estimated 5-year survival rate of 39% (Jemal et al., 2004). During diagnosis, 60% of patients present with advanced stage of the disease (Munkarah and Coleman, 2004). Ovarian peritoneal carcinomatosis (OPC) is considered the terminal stage of the disease and consists of macroscopic tumor nodules of variable sizes and consistencies that can coalesce to form plaques or masses within the abdominopelvic cavity. Comprehensive management using surgical cytoreduction and intraperitoneal chemotherapy can improve the quality of life and survival of patients. Imaging evaluation of patients with OPC using multidetector computed tomography (MDCT) or MRI (MRI) is limited for the assessment of progression or stability of the disease as there are no well-established and standardized criteria (Eisenhauer et al., 2009; Wasnik et al., 2015). Implants of OPC are distributed in the abdominopelvic cavity according to the circulation of the peritoneal fluid (Eisenhauer et al., 2009). The blood flow supply of the abdominopelvic cavity depends on the superior mesenteric artery (SMA) and the coeliac trunk (CT). The SMA supplies the mesentery, the visceral peritoneum, the lower part of the duodenum, the transverse colon, and the pancreas. The CT supplies the stomach, the liver, the spleen, the diaphragmatic cupolas, the upper duodenum, and the pancreas.

### Pseudomyxoma Peritonei

Pseudomyxoma peritonei is a rare malignant disease characterized by the progressive accumulation of mucins in the peritoneal cavity and by the diffusion of ascites without extraperitoneal diffusion, leading to compression of the intra-abdominal organs and a fatal outcome (Smeenk et al., 2008). The consensus is that PMP has an intestinal origin and results from the perforation of a mucinous appendiceal neoplasm (Cuatrecasas et al., 1996; Guerrieri et al., 1997; Ronnett et al., 1997; Szych et al., 1999). With a mouse model of orthotopic xenograft of mucinous implants, PMP was demonstrated to present low cellularity but sustained tumor angiogenesis grafted on the native vascular network of the peritoneal layers mainly supplied by the SMA (Dohan et al., 2014). In human, implants of PMP are distributed in the abdominal cavity with nodules grafted on the surface of abdominopelvic organs supplied by the SMA and by the CT (Figure 2). The curative treatment combines complete cytoreductive surgery and hyperthermic intraperitoneal chemotherapy. This treatment imposes a clinical and radiological follow-up in order to identify an abdominal recurrence that can be used to conduct a second surgical intervention and/or a systemic chemotherapy.

The article "Blood Flow and Shear Stress Allow Monitoring of Progression and Prognosis of Tumor Diseases" was published in 2021. Journal: Front Physiol.

**Figure 2:** Schematic representation of hemodynamic modifications in the superior mesenteric artery (SMA) during the development of a peritoneal carcinomatosis (PC). **(A)** In healthy conditions, SMA supplies the bowel and the mesentery. **(B)** Blood flow velocity waveform recorded in the SMA after an overnight fast, the bowel and mesentery vascular network set the mean blood flow velocity BFVel), and the blood flow volume (BFVo to normal values (17.2 cm/s, 232 ± 50 mL/min respectively), the SMA inner diameter and the BFVel are well-balanced to maintain the WSS in normal ranges (8.7 ± 2.8 dynes/cm^2^). **(C)** In the case of PC, an abnormal tumor vascular network develops from the native vascular network. **(D)** Shows a representative bidimensional ultrasound horizontal cross-sectional view illustrative of the expansion of the disease into the whole abdominal cavity. **(E)** Corresponding increased BFVel recorded in the SMA (BFVel: 34.3 cm/s), the inner diameter is not increased but the BFVol is increased (525 mL/min) corresponding to the progressive disease. **(F)** In patients with pseudomyxoma peritonei (PMP), the BFVol increases in the SMA proportionally to the per-operative peritoneal carcinomatosis index (PCI).

### Superficial Arteriovenous Malformation

Facial superficial AVMs are rare and may significantly impair the quality of life of patients because of their esthetic prejudice. AVMs are vascular malformations composed of arteries that directly communicate with veins through a central “nidus.” The absence of the high resistive arterioles of a normal microvascular network induces a drop in vascular impedance with high flows and without any vasomotor regulation that shunts blood from the arterial to the venous sides of the local circulation with the appearance of an early venous return. Therefore, superficial AVMs are responsible for a significant and permanent increase of the blood flows in the upstream native conduit arteries; the levels reached by the BFVols in these upstream native arteries depend on the size of the downstream vascular lesion. The curative treatment combines the complete resection of the vascular lesion or interventional radiology procedures, including embolization or percutaneous cryotherapy (Dubois and Alison, 2010; Cornelis et al., 2013; Mulligan et al., 2014). However, these treatments may result in complications and morbidity, and the decision for invasive management should be carefully balanced. The timing of treatment remains debated: (1) resection when performed too late leads to large excision and disfigurement, (2) embolization aiming to occlude the nidus, when incomplete, can secondarily stimulate the development of the vascular lesion, (3) both can lead to extended tissue loss with major esthetic damages and disfiguration when located on the face. While stable superficial AVM may be managed conservatively with scheduled clinical and radiological follow-ups, a therapeutic window is usually considered for surgical treatment of progressive superficial AVM (Lee et al., 2013; Morgan et al., 2016). Thus, the assessment of the aggressiveness of the lesion is crucial to determine the most appropriate strategy and to avoid iatrogenic complications. The progression of the disease is usually assessed by composite parameters, including clinical changes on successive examinations and increases of the blood flow in the afferent arteries associated with the expansion of the nidus on Doppler ultrasound recordings, magnetic resonance angiography (MRA), and conventional angiograms. Consequently, changes in BFVol have been previously suggested as a biomarker of disease progression in AVM (Uller et al., 2014).

The article "Blood Flow and Shear Stress Allow Monitoring of Progression and Prognosis of Tumor Diseases" was published in 2021. Journal: Front Physiol.

## Patients and Methods

### Patients With OPC, Preoperative Doppler Ultrasound Evaluation

After IRB approval (ID GRIVIL 09-11-016) and obtaining informed consent from patients, 21 women aged 53 ± 30 [30–74] years were included and had Doppler ultrasound a few days before cytoreductive surgery and hyperthermic intraperitoneal chemotherapy (1.7 ± 1.0 months) from May 1, 2016 to April 30, 2019. All patients underwent peritoneal laparoscopy during the cytoreductive surgery and the per-operative peritoneal carcinomatosis index (PCI) [13 ± 12 (1–39)] was determined 16.0 ± 18.5 months after OPC diagnosis.

### Patients With PMP, Preoperative and Postoperative Doppler Ultrasound Evaluation

After institutional review board (IRB) approval (ID GRIVIL 09-11-016), and obtaining informed consent from patients, patients were included when they were scheduled to undergo cytoreductive surgery or after surgery for PMP from October 1, 2011 to October 1, 2020. The cohort was partly previously described in studies aiming to determine the changes in BFVels, arterial diameters, BFVols, and WSS in the SMA (52 patients) (Dohan et al., 2017; Barral et al., 2019). This cohort of patients now includes 128 patients (68 patients with preoperative Doppler ultrasound examination, 1.1 ± 0.9 months before surgery, and 60 with postoperative Doppler ultrasound examination, 17.3 ± 10.0 months after surgery). All patients had a peritoneal exploration with determination of the PCI during cytoreductive surgery. The completeness of cytoreductive surgery determined the decision to perform hyperthermic intraperitoneal chemotherapies (Sugarbaker and Jablonski, 1995; Jacquet and Sugarbaker, 1996). All patients had a pathological analysis with an evaluation of the tumor grade according to the WHO classification (Carr et al., 2012).

The article "Blood Flow and Shear Stress Allow Monitoring of Progression and Prognosis of Tumor Diseases" was published in 2021. Journal: Front Physiol.

For preoperative Doppler ultrasound evaluation, patients were distributed into two groups according to their clinical outcome. Completeness of resection was graded according to complete cytoreduction (CCR) score of Sugarbaker as follows: CCR0: no residual tumor; CCR1: residual tumor with nodules < 0.25 cm; CCR2: residual tumor between 0.25 and 2.5 cm; CCR3: residual tumor with tumor nodules > 2.5 cm (Glehen et al., 2004). ***Group-A***included 33 patients with complete resection (CCR0) and hyperthermic intraperitoneal chemotherapy, without any recurrence within 3 years after surgery. ***Group-B***included 35 patients with incomplete resection (CCR1, CCR2, or CCR3 score). Characteristics of patients are reported in Table 1.

**Table 1:** Preoperative study, pseudomyxoma peritonei, and characteristics of patients.

	**Controls (*n* = 24)**	**Group-A (CCR0) (*n* = 33)**	**Group-B (CCR1-2-3) (*n* = 35)**	***X*^**2**^ test *p-*value**	**One-way ANOVA (between Cont., GA, GB, or between GA, GB)**
**Age (years)**					
Mean (SD)	43 (13)	58^*^ (13)	59^*^ (12)		Cont., G-A, G-B: *p* < 0.001,
[range]	[22–69]	[26–76]	[34–87]		G-A vs. G-B: *p* = 0.032
**Gender [Patients (** ***n*** **)]**					
Women	10	22	9	0.079	-
Men	14	11	26		
**Per-operative PCI**					
Mean	-	14	30^##^		0.002
(SD)		9	7		
[range]		[1–34]	[30–39]		
**Postoperative PCI**					
Mean	-	0	25^##^		
(SD)		0	10		
[range]			[1–39]		
**Grade [Patients (** ***n*** **)]**					
Low	-	25	24	0.193	-
High		8	11		
**Delay between diagnosis and surgery (years)**					
Mean (SD)	-	1.6 (2.9)	1.3 (2.5)		0.126
[range]		[0.1–10.1]	[0.1–11.3]		

*SD, standard deviation; PCI, Peritoneal Cancer Index at surgery; CCR, complete cytoreduction score*.

* *p < 0.005 vs. controls*.

## *p < 0.001 vs. group-A*.

*-, not applicable*.

For postoperative Doppler ultrasound evaluation, patients were distributed into three groups according to their clinical outcome. ***Group-1***included 24 patients with complete resection (CCR0) and hyperthermic intraperitoneal chemotherapy without any recurrence within 3 years after surgery. ***Group-2***included 22 patients; these patients had incomplete resection (CCR1, CCR2, or CCR3 score) and slowly progressive disease: still alive 3 years after the surgery or at least during follow-up without disease progression (i.e., progression free). ***Group-3***included 14 patients; these patients had incomplete resection (CCR1, CCR2, or CCR3 score) with progressive disease. Progression corresponded to patients with performance status>1 or dead within 3 years after the surgery. The onset of new mucinous deposit on MDCT or MRI within 6 months after surgery was considered as a progression (recurrence). All patients had serum tumor markers measurements of carcinoembryonic antigen (CEA) and carbohydrate antigen 19-9 (CA 19-9) at the same time of Doppler ultrasound (not shown). Adult healthy patients were also enrolled as controls (*n* = 24). Characteristics of patients are reported in Table 2.

The article "Blood Flow and Shear Stress Allow Monitoring of Progression and Prognosis of Tumor Diseases" was published in 2021. Journal: Front Physiol.

**Table 2:** Postoperative study, pseudomyxoma peritonei, and characteristics of patients.

	**Controls (*n* = 24)**	**Group-1 (CCR0-1, stable) (*n* = 24)**	**Group-2 (CCR2-3, stable) (*n*= 22)**	**Group-3 (CCR2-3, progression) (*n* = 14)**	***X*^**2**^ test *p-*value**	**One-way ANOVA (between Cont., G1, G2, G3, or between G1, G2, G3)**
**Age (years)**						
Mean (SD)	43 (13)	56 (13)	60^*^ (10)	65^**^ (12)		Cont., G1, G2, G3: *p* < 0.001
[range]	[22–69]	[33–78]	[52–73]	[46–87]		G1, G2, G3: *p* = 0.032
**Gender [Patients (** ***n*** **)]**						
Women	10	13	6	8	0.242	-
Men	14	11	16	6		
**Per-operative PCI**						
Mean	-	18	27^#^	29^#^		0.002
(SD)		10	11	4		
[range]		[1–30]	[4–39]	[24–36]		
**Postoperative PCI**						
Mean	-	0	11^##^	22^##^		0.001
(SD)		0	16	10		
[range]			[1–39]	[1–29]		
**Grade [Patients (** ***n*** **)]**						
Low	-	18	15	8	0.366	-
High		6	7	6		
**Delay between diagnosis and surgery (years)**						
Mean	-	3.0	1.3	2.3		0.004
(SD)		(4.5)	(2.5)	(4.5)		
[range]		[0.1–10.1]	[0.2–4.2]	[0.1–3.3]		
**Postoperative chemo therapy [Patients (** ***n*** **)]**						
Yes	-	0	2	2	0.088	-
No		0	0	0		
**Postoperative bevacizumab [Patients (** ***n*** **)]**						
Yes	-	0	1	1	0.516	-
No		0	0	0		

*SD, standard deviation; PCI, Peritoneal Cancer Index at surgery; CCR, complete cytoreduction score*.

* *p < 0.005*,

** *p < 0.001 vs. controls*.

# *p < 0.005 vs. group-1*.

## *p < 0.001 vs. group-1*.

*-, not applicable*.

### Patients With SAM, Preoperative, and Postoperative Doppler Ultrasound Evaluation

After IRB approval (ID RCB 2015AO 177-42) and obtaining informed consent from patients, 110 patients were included from January 1, 2017 to October 30, 2020. The cohort was previously partly described in a study aiming to determine the modifications of the blood flows, arterial diameters, and WSS in facial superficial AVM (40 patients) (El Sanharawi et al., 2020). The cohort now comprises patients with (1) complete resected lips, cheek, mandible, ear, scalp, and forehead superficial AVM (*n* = 44) and (2) active superficial AVM of the same localization under active surveillance (*n* = 66). Pregnant women and children were excluded. Healthy adult patients were enrolled as controls (*n* = 15).

The article "Blood Flow and Shear Stress Allow Monitoring of Progression and Prognosis of Tumor Diseases" was published in 2021. Journal: Front Physiol.

All patients had a clinical examination, at inclusion and after 6 months, blinded from the sonographer. According to the Schobinger classification, patients were classified as follows: stage 1: quiescent; stage 2: expansion; stage 3: destruction; and stage 4: decompensation (Kohout et al., 1998). Patients were distributed into three groups: ***group-1***: operated patients with complete resection of the superficial AVM at least 6 months before Doppler ultrasound examination, without any clinical sign of recurrence (*n* = 44); ***group-2***: patients with stable clinical and radiological superficial AVM for more than 1 year (*n* = 26); ***group-3***: patients with clinical active progressive superficial AVM (*n* = 40). Stage 1 or 2 AVM was considered as stable. Progressive AVM was defined as a growing AVM on two consecutive clinical examinations following Doppler ultrasound examination and blinded from Doppler results or when classified in Schobinger stage 3 or 4. All patients underwent bilateral common, internal, external carotid, facial, and/or superficial temporal arteries (STAs) Doppler ultrasound. Characteristics of patients are reported in Table 3.

**Table 3:** Arteriovenous malformation and characteristics of patients.

	**Controls (*n* = 15)**	**Group-1 (operated AVM) (*n* = 44)**	**Group-2 (stable AVM) (*n* = 26)**	**Group-3 (progressive AVM) (*n* = 40)**	***X*^**2**^ test *p-*value**	**One-way ANOVA (between Cont., G1, G2, G3, or between G1, G2, G3) *p-*value**
**Age (years)**						
Mean (SD)	44 (13)	37 (14)	36 (13)	32 (13)		Cont., G1, G2, G3: *p* = 0.043
[range]	[24–62]	[18–75]	[22–59]	[20–50]		G1, G2, G3: *p* = 0.219
**Gender [Patients (** ***n*** **)]**						
Female	9	30	13	28	0.170	
Male	6	14	13	12		
**AVM location**						
	-	Lip: 19 Nose: 3 Cheek: 5 Mandible: 3 Forehead: 3 Ear: 6 Scalp: 5	Lip: 7 Nose: 1 Cheek: 3 Mandible: 3 Forehead: 5 Ear: 2 Scalp: 2	Lip: 12 Nose: 1 Cheek: 11 Mandible: 5 Forehead: 7 Ear: 6 Scalp: 0	0.287	
**Schobinger stage at the beginning of the study**						
	-	-	Stage 1: 0 Stage 2: 26 Stage 3: 0 Stage 4: 0	Stage 1: 0 Stage 2: 40 Stage 3: 0 Stage 4: 1		
**Schobinger stage at the end of the study**						
	-	-	Stage 1: 0 Stage 2: 26 Stage 3: 0 Stage 4: 0	Stage 1: 0 Stage 2: 36 Stage 3: 3 Stage 4: 1		
**Familial history of AVM**						
	-	0	0	0		
**Duration between surgery and Doppler exam (months)**						
Mean (SD)	-	42 (41)	-	-		
[range]		[7–125]				

*SD, standard deviation; AVM, arteriovenous malformation*.

*-: not concerned*.

The article "Blood Flow and Shear Stress Allow Monitoring of Progression and Prognosis of Tumor Diseases" was published in 2021. Journal: Front Physiol.

### Doppler Ultrasound Studies

All Doppler ultrasound examinations were performed with an ultrasound apparatus ACUSON S2000 (Siemens, Erlangen, Germany) equipped with a linear transducer type CH4-1 (3.5 MHz) for digestive arteries examination as previously described (Bonnin et al., 2013), with a linear transducer type L (12–7.5 MHz) for common carotid artery (CCA) and external carotid artery (ECA) and with a linear transducer type L (18.8 MHz) for facial arteries (FA) or STAs.

#### Superior Mesenteric Artery Doppler Ultrasound Examination

Doppler ultrasound was performed in patients and controls in a hemi-seating position to get access to the SMA at its first centimeters. The examination was performed after an overnight fast to avoid variations in the blood flows occurring during digestion and with an empty stomach to avoid gas interposition above the SMA. The SMA was studied in the long axis using an anterior sagittal cross-sectional view of the abdomen. Color-coded Doppler ultrasound was activated for recognition of digestive arteries in front of the aorta then switched off. M-mode was first activated for measurements of systolic and diastolic inner diameters of the SMA. Steer mode was used to ensure measurement of the diameters strictly perpendicular to the longitudinal axis of the artery with the placement of the calipers at the intimal borders of the artery. The ultrasound transducer was then displaced and adequately oriented to improve the angle between the Doppler beam and the longitudinal axis of the artery, the best of which would be inferior to 35–45°. Pulsed Doppler ultrasound was secondly activated for BFVel waveforms acquisition with the positioning of the sample volume on the SMA about 2–3 cm after its origin but proximal to any side branches, with adjustment of the sample volume to the whole arterial section (Figures 2B,E, 3). A cutoff filter of 100 to150 Hz was applied to exclude artifacts from vessel wall motion. Great care was taken for angle correction adjustment anyway below 60° to calculate true velocities.

**Figure 3:** **(A)** Bidimensional longitudinal cross-sectional view of the aorta (Ao), the coeliac trunk (CT), and the SMA permitting to place the line for M-mode strictly orthogonal to the longitudinal axis of the artery. **(B)** M-mode activation on the SMA permits to place calipers to measure systolic and diastolic inner diameters and to calculate the mean diameter (here, 0.61 cm). **(C)** Doppler spectral analysis of the blood flow velocity waveform recorded in the SMA; the blue line represents the instantaneous mean blood flow velocity (BFVel = 18.5 cm/s) obtained after application of the angle-correction between the Doppler beam and the longitudinal axis of the artery (41°). The BFVo) is then calculated (324 mL/min).

The article "Blood Flow and Shear Stress Allow Monitoring of Progression and Prognosis of Tumor Diseases" was published in 2021. Journal: Front Physiol.

#### Common, External Carotid, and Facial Arteries Doppler Ultrasound Examination

Doppler ultrasound was performed at rest in a supine position in both ipsilateral and contralateral CCA, ECA, and FA or STA in patients and controls. Arteries were first recognized and visualized in a long axis with color-coded Doppler. M-mode was used to measure inner diameters; pulsed Doppler ultrasound was activated for BFVel waveforms acquisition. Great care was taken for angle correction adjustment anyway below 60° to calculate true velocities.

#### For All Arteries

For all arteries, peak systolic, end diastolic, time-average maximal (max-BFVel), and spatial-average-time-average (mean-BFVel) velocities were measured from the spectral analysis of the Doppler BFVel waveforms. The max-BFVel is a computer-derived value calculated by integrating all the areas under envelope of the waveform. The mean-BFVel is the computed-derived value calculated by integrating the area under instantaneous mean velocity. Indeed, BFVel profile is parabolic in peripheral vessels, thus total displacement of blood is represented by the displacement of all the layers of blood on the arterial section, not only the highest one in the center of the arterial section but also of the lower ones near the arterial wall. The mean-BFVel is representative of the mean blood displacement over the whole arterial section and over the cardiac cycle per time unit.

Blood flow volume (BFVol) must be calculated with mean-BFVel following the formula:

BFVol = π. r^2^. mean-BFVel.60

where BFVol is the blood volume in mL/min, mean-BFVel is the spatial-averaged-time-averaged mean BFVel in cm/s, and r is the radius of the artery in cm (Collins et al., 2003). Each measurement was taken in triplicate during quiet respiration and averaged.

Wall Shear stress is calculated following the formula:

τ = 4.μ.BFVol/π.r^3^ or τ = 8.μ. mean-BFVel /d

where τ is the WSS in dynes/cm^2^, μ is the blood viscosity in poise (P), mean-BFVel is the spatial-averaged-time-averaged BFVel (cm/s), and d is the diameter (cm). In conduit arteries, blood acts like a Newtonian fluid, and a viscosity value of 0.035 P can be used to calculate the WSS; the normal value for WSS ranges around 8–10 in conduit arteries to 50 dynes/cm^2^ in the arterioles (Papaioannou and Stefanadis, 2005). Hematocrit and total plasma proteins concentrations are two factors that can influence the value of viscosity. An analysis of covariance was performed on the WSS calculated with a fixed viscosity of 0.035 P between patients with PMP with stability or progression of their disease including confounding factors Hematocrit and total plasma proteins concentrations measured at the time of the Doppler study. No interference was found on the WSS values between the different groupw (*p* = 0.551), which can be attributed to the individual Hematocrit (*p* = 0.286) or of total plasma proteins concentrations (*p* = 0.286), allowing to avoid paying attention to the level of biological parameters to evaluate the WSS with a generic viscosity of 0.035 P for clinical use.

The article "Blood Flow and Shear Stress Allow Monitoring of Progression and Prognosis of Tumor Diseases" was published in 2021. Journal: Front Physiol.

### Statistics

Results are presented as mean ± SD [Min-Max]. The BFVols measured in SMA were correlated to the PCI using a Pearson's test for patients with OPC or PMP. In AVMs, as the FAs and the STAs presented identical inner diameters in controls (NS) and supply similar bone-muscle-skin territories, the Doppler ultrasound results of the FA or of the STA were pooled. One-way ANOVAs were applied to compare values between patients and healthy controls. *Post-hoc* Student-Newman-Keuls were performed to differentiate between groups. A receiver operating characteristics (ROC) curve for mean-BFVel, BFVols, and WSS were built, and a cutoff value was calculated to discriminate between patients without from those with progressive disease. Areas under curves (AUC) were calculated and optimal cutoffs were obtained by maximizing Youden index to reach the best balance between sensitivity and specificity-1 (MedCalc^®^ Statistical Software version 18.2.1, MedCalc Software bvba, Ostend, Belgium). As no gender or age effects were found on diameters, BFVels, BFVols, or WSSs in PMP or AVM studies, all data were pooled in each group. The degree of significance of the selected tests was *p* < 0.005 (Johnson, 2013). For all patients, the treatment was not driven by Doppler ultrasound findings, and the clinical practitioner or the surgeon was blind to these Doppler ultrasound results.

## Results

### Blood Flow Volume Reflects Tumor Burden in OPC and PMP

In preoperative settings, patients with OPC had superior BFVols than healthy controls [377 ± 110 (223–585) and 231 ± 51 (117–323) mL/min, respectively, *p* < 0.001]. BFVol measured before cytoreductive surgery was correlated to the per-operative PCI as shown by a positive linear regression (*n* = 21, *R*^2^ = 0.6236, *p* < 0.001). Patients with PMP also presented increased BFVols [397 ± 193 (151–960) mL/min, *p* < 0.001 vs. controls]. A positive linear regression between preoperative BFVol and PCI was found (*n* = 66, *R*^2^ = 0.4028, *p* < 0.001, Figure 2F). Moreover, patients with a CC0 score, i.e., those with a relatively low preoperative tumor burden [PCI = 18 ± 8 (2–34)] exhibited a preoperative BFVol of 338 ± 124 (151–616) mL/min, similar to normal values, although patients with a CC123 score, i.e., those with a relatively high tumor burden [PCI = 27 ± 10 (13–39), *p* = 0.0274 vs. CC0 patients] presented high preoperative BFVol (567 ± 197 mL/min, *p* < 0.001 vs. CC0 patients, *p* < 0.001 vs. controls).

The article "Blood Flow and Shear Stress Allow Monitoring of Progression and Prognosis of Tumor Diseases" was published in 2021. Journal: Front Physiol.

In the postoperative settings, BFVol decreased in group-1 18.0 ± 14.4 months after surgery to 267 ± 103 [128–274] mL/min (NS vs controls) while it remained elevated in group-2 to 417 ± 158 [165–763] (*p* < 0.001 vs controls and group-1) and group-3 to 600 ± 193 [375–1,035] mL/min (*p* < 0.001 vs. controls, group-1, and group-3) consistent with the increase in tumor burden, thus recurrence (Table 4). Recurrence was consistently evidenced on MDCT and/or MRI 29.0 ± 14.3 in group-2 and 20.9 ± 12.7 months in group-3 after surgery, i.e., a few months after performance of the Doppler ultrasound.

**Table 4:** postoperative hemodynamics in patients with PMP, hemodynamics in patients with AVM.

	**Inner diameter**	**Mean BFVel**	**BFVol**	**WSS**	**Cutoff**
	**(cm)**	**(cm/s)**	**(mL/min)**	**(dynes/cm^**2**^)**	**(dynes/cm^**2**^)**
**PSEUDOMYXOMA PERITONEI**					
**Superior mesenteric artery**					
**Controls (** ***n*** **=** **24)**	0.54 ± 0.06	16.9 ± 4.8	232 ± 50	8.7 ±−2.8	
**Group-1**					
Resection completed (*n* = 24)	0.55 ± 0.09	18.9 ± 4.0	267 ± 103	9.9 ± 2.7	
**Group-2**					
Stable disease (*n* = 22)	0.64 ± 0.06^***^	20.8 ± 4.8	**417** ± 158^***^	9.2 ± 1.7	
**Group-3**					**12.1**
Progressive disease (*n* = 14)	0.56 ± 0.08^##^	38.4 ± 12.8^***^, *^###^*	**600** ± 193^***^, *^###^*	19.6 ± 7.9^***^, *^###^*	
**FACIAL ARTERIOVENOUS MALFORMATION**					
**Common carotid artery (ipsilateral)**					
**Controls (** ***n*** **=** **15)**	0.55 ± 0.08	20.6 ± 4.8	292 ± 64	10.7 ± 3.3	
**Group-1**					
Resection completed (*n* = 44)	0.56 ± 0.07	21.7 ± 3.9	328 ± 94	11.0 ± 2.5	
**Group-2**					
Stable disease (*n* = 26)	0.64 ± 0.10^***^	22.1 ± 4.5	**435** ± 167^***^	9.8 ± 2.5	
**Group-3**					**9.5**
Progressive disease (*n* = 40)	0.61 ± 0.11	27.5 ± 5.7^***^, *^###^*	**510** ± 342^***^	12.8 ± 2.6^***^, *^###^*	
**External carotid artery (ipsilateral)**					
**Controls (** ***n*** **=** **15)**	0.43 ± 0.07	14.3 ± 4.0	120 ± 40	8.6 ± 2.2	
**Group-1**					
Resection completed (*n* = 44)	0.42 ± 0.08	15.6 ± 4.0	136 ± 64	10.5 ± 3.0	
**Group-2**					
Stable disease (*n* = 26)	0.51 ± 0.11^***^	18.7 ± 4.8^***^	**237** ± 115^***^	10.7 ± 3.1	
**Group-3**					**12.1**
Progressive disease (*n* = 40)	0.48 ± 0.11	24.7 ± 9.6^***^, *##*	**313** ± 318^***^	14.2 ± 3.8^***^, *^###^*	
**Afferent artery (ipsilateral)**					
**Controls (** ***n*** **=** **15)**	0.16 ± 0.03	10.9 ± 2.8	13 ± 6	20.3 ± 6.1	
**Group-1**					
Resection completed (*n* = 44)	0.16 ± 0.04	11.7 ± 4.6	14 ± 8	21.5 ± 8.2	
**Group-2**					
Stable disease (*n* = 26)	0.24 ± 0.08^***^	17.5 ± 6.4^***^	**62** ± 49^***^	20.8 ± 4.3	
**Group-3**					**26.5**
Progressive disease (*n* = 40)	0.19 ± 0.06^**^, *^###^*	30.5 ± 13.3^***^, *^###^*	**63** ± 62^***^	46.4 ± 6.5^***^, *^###^*	

*Afferent artery: facial or superficial temporal artery depending on the location of the nidus on the face*.

The article "Blood Flow and Shear Stress Allow Monitoring of Progression and Prognosis of Tumor Diseases" was published in 2021. Journal: Front Physiol.

***In bold**: persistent disease, **in red color**: achieved expansive arterial remodeling (normalized WSS) permitting recognition of a stable disease, **in blue color**: absence of achieved arterial remodeling permitting the recognition of a progression disease (Mean ± Standard Deviation*,

** *p < 0.005*,

*** *p < 0.001 vs. controls*,

## *p < 0.005*,

### *p < 0.001 progressive vs. stable disease)*.

### WSS Evaluates Disease Progression

#### Preoperative WSS in OPC and PMP

Preoperative WSS calculated in the SMA of women with OPC was higher than controls at one time point [15.2 ± 7.2 (6.5–35.7) and 8.7 ± 2.8 (5.0–13.3) dynes/cm^2^ respectively, *p* < 0.001]. Preoperative WSS was similar in CC0 and CC123 patients with PMP, 11.2 ± 4.4 (5.6–20.8) and 14.0 ± 6.5 (5.6–32.8) dynes/cm^2^ (NS), respectively, but both were superior to the values of controls (*p* < 0.001, both). Preoperative WSS thus suggested a continuous expansion of the disease. However, preoperative WSS was not predictive of the long-term outcome after treatment in women with OPC.

#### Postoperative WSS in PMP

Postoperative WSS determined 1 year after surgery remained normal at 9.9 ± 2.7 (4.3–16.5) dynes/cm^2^ in group-1 patients (NS vs. controls). Group-2 patients presented a WSS of 9.2 ± 1.7 (5.7–12.1) dynes/cm^2^ (NS vs. group-1 patients, NS *vs* controls), although the BFVol remained elevated at 414 ± 158 (165–763) mL/min, indicative of a persistent tumor burden. BFVels and WSS normalized because of an achieved arterial remodeling of the SMA during the year following the cytoreductive surgery revealed by an actual increase in the inner diameter of SMA [0.64 ± 0.06 (0.49–0.76) cm, *p* < 0.001 vs. controls, *p* < 0.001 vs. group-1, *p* < 0.001 vs. group-3] (Table 4). Arterial remodeling in humans is a delayed process that needs a few months to reach a balance between arterial inflow and the downstream vascular network, followed by normalization of the WSS in the artery plaids in favor of the stability of the tumor burden during the year following the cytoreductive surgery. Normalization of the WSS was observed only in patients with clinical and radiological slowly progressive status (group-2). Conversely, in group-3 patients i.e., with incomplete resection and active progressive disease, the BFVols were dramatically augmented, illustrative of an increase in the tumor burden. Moreover, the absence of any achievement of arterial remodeling in the afferent artery, the SMA, illustrated by the persistence at 1 year of elevated BFVels and WSS and lower inner diameter of the SMA [0.56 ± 0.08 (0.49–0.72) cm, *p* < 0.005 vs. group-2 patients, NS vs. controls and group-1 patients], leads to a progression of the disease during the year following the cytoreductive surgery. The use of the WSS permitted to differentiate group-3 from group-1 and−2 [ROC-curve analysis, AUC = 0.978 (95% CI: 0.902–0.999), *p* < 0.0001] with a sensitivity of 100.0%, a specificity of 93.5%, and a cutoff of >12.1 dynes/cm^2^ (Figures 4A, 5). The use of the BFVels permitted to differentiate group-3 from group-1 and−2 with a slightly less sensitivity and specificity [AUC = 0.948 (0.883, 0.996), *p* < 0.0001, sensitivity: 92.9%, specificity: 93.5%, cutoff: 25.0 cm/min] (Figure 4B); the use of the BFVol permitted to differentiate group-3 from group-1 and−2 [AUC = 0.866 (95% CI: 0.753, 0.940), *p* < 0.0001, sensitivity: 100.0%, specificity: 63.8%, cutoff >365 mL/min] (Figure 4C).

The article "Blood Flow and Shear Stress Allow Monitoring of Progression and Prognosis of Tumor Diseases" was published in 2021. Journal: Front Physiol.

**Figure 4:** ROC curves analysis of **(A)** the wall shear stress (WSS), **(B)** the mean blood flow velocity BFVel, **(C)** the BFVol recorded in the SMA. Calculation of the cutoffs permits to differentiate slowly from active (recurrence) progressive PMP 1 year after a cytoreductive surgery (± hyperthermic intraperitoneal chemotherapy).

**Figure 5:** WSS calculated in the SMA 1 year after postoperative in patients with PMP. *Group-1* patients with complete resection (CCR0) without any recurrence within 3 years after surgery; the WSS normalized and was identical to WSS in *controls*. *Group-2* patients with persistent and slowly progressive disease after surgery, with arterial remodeling processes of the SMA achieved and the WSSs normalized. G*roup-3* patients with persistent and active progressive disease (recurrence), with the WSSs dramatically increased beyond a cutoff of 12.1 dynes/cm^2^.

#### WSS in Arteriovenous Malformation

In AVM disease, patients with successful resection of the nidus (group-1) presented similar inner diameters, BFVels, BFVols, and WSS in the CCA, ECA, and the afferent artery than controls during the Doppler ultrasound examination performed at least 6 months after surgery. Patients with clinical and radiological stability of their disease (group-2) presented similar high BFVols in the afferent arteries than group-3 patients with the progressive disease with clinical and radiological progression during the 6 months preceding the Doppler ultrasound examination. Nevertheless, the BFVels and the WSS were normal in group-2 patients consecutive to the achievement of the remodeling processes evidenced by higher inner diameters of all afferent arteries, although they were elevated in group-3 patients consecutive to the absence of any arterial remodeling achievement (Table 4). The use of the WSS in CCA, ECA, and the afferent artery permitted to differentiate group-3 from group-2 patients with higher performance when Doppler ultrasound was performed closer to the vascular lesion, sensitivity: 93.9, 81.2, 93.5%, specificity: 55.6, 77.8, 95.8%, respectively, in ipsilateral CCA, CEA, and the afferent artery (*p* < 0.0001 in all arteries, ROC-curves analysis) (Figures 6A–C). The highest sensitivity and specificity of WSS in the afferent arteries can be attributed to the proximity of the vascular lesion thus the arteries with the more important load effect. The cutoffs scaled from >9.5 to >12.1 and >26.5 dynes/cm^2^, respectively, in the ipsilateral CCA to the ECA and the closer afferent artery (Figures 6A–C, 7).

The article "Blood Flow and Shear Stress Allow Monitoring of Progression and Prognosis of Tumor Diseases" was published in 2021. Journal: Front Physiol.

**Figure 6:** ROC curves analysis of the wall shear stress recorded in the ipsilateral afferent arteries, upstream an arteriovenous malformation of the face. **(A)** Common carotid, **(B)** external carotid, **(C)** closer afferent arteies, i.e., in the facial or superficial temporal artery. The WSS calculated closer to the vascular lesion permits to differentiate the patients with stable disease from those with active progressive disease. The elevation of the WSSs is illustrative of the imbalance between the afferent arteries and the vascular lesions in expansion, although a normal WSS is representative of the stability of the lesion. The hemodynamic status in the afferent artery permits the recognition of the progression of the disease. Sensitivity and specificity increase the closer the explored artery is to the vascular due to the mass effect of the BFVol dedicated to supplying the vascular lesion on the normal BFVol.

**Figure 7:** WSS calculated in the closer contralateral or ipsilateral afferent arteries, facial, or superficial temporal arteries, of patients with a facial superficial AVM. In operated patients *(group-1)*, the WSS normalized and was identical to WSS in *controls*. In patients with stable disease (*group-2*), arterial remodeling processes were achieved and the WSSs was normalized. In patients with progressive disease *(group-3)*, the WSSs dramatically increased beyond a cutoff of 26.5 dynes/cm^2^ in the ipsilateral afferent artery. The WSS was also elevated in group-3 patients in the contralateral afferent artery due to its participation in perfusion of the lesion through the side-to-side anastomoses particularly developed in the subcutaneous tissues of the face.

The article "Blood Flow and Shear Stress Allow Monitoring of Progression and Prognosis of Tumor Diseases" was published in 2021. Journal: Front Physiol.

## Discussion

Development of pathological vascular networks characterizes OPC, PMP, and AVM. However, in those diseases, progression remains difficult to predict (Sun et al., 2009; Carr et al., 2012; Lee et al., 2013; Morgan et al., 2016). The growth of the vascular network is responsible for a drop in vascular impedance with a consecutive increase in blood flows of afferent native conduit arteries, with an upstream in the organs where the tumor vascular networks develop. This induces marked upstream hemodynamic changes in the afferent arteries driven by the increase in BFVol and, particularly in WSS, inducing the arterial remodeling processes. Therefore, measurement of the BFVols in the SMA just before cytoreductive surgery in patients with OPC and PMP appears predictive of the tumor burden. Moreover, measurement of the WSS in patients with PMP at 1 year after cytoreductive surgery and in patients with AVM permits in identifying disease progression with high sensitivities and specificities with cutoffs of 12.1 dynes/cm^2^ in the SMA and the ECA and of 26.5 dynes/cm^2^ in the FA and STA.

Several experimental studies were previously performed to test the hypothesis of blood flow increase during tumor angiogenesis. Monitoring of the BFVels in the afferent arteries of injured organs permits to follow quantitatively the tumor angiogenesis in mouse models of spontaneous hepatocellular carcinoma (HCC) and of PC with orthotopic tumor allograft or xenograft. In those studies, only BFVels were monitored using Doppler ultrasound examination because of the absence of sufficient accuracy of measurement of inner diameters of the afferent arteries in the mouse. Efficacy of antitumor therapies in HCC murine models (Bonnin et al., 2007; Vincent et al., 2009; Bergé et al., 2010; Eveno et al., 2012; Barral et al., 2016) and of procedures of cytoreductive surgery coupled with antitumor therapies in PMP was monitored by assessment of BFVels (Dohan et al., 2014; Lo Dico et al., 2018; Barral et al., 2021). In human, changes in BFVol have been previously suggested as a biomarker of disease progression in patients with PMP and AVM (Uller et al., 2014; Dohan et al., 2017). In patients with PMP, BFVol measured in the SMA 1 year after surgery was able to predict tumor progression (Dohan et al., 2017). In patients with a facial superficial AVM, only augmentations in BFVol measured in the upstream native arteries by Doppler ultrasound between two successive examinations until now allow the monitoring of AVM progression (Mulligan et al., 2014). Quantitative evaluation of the extension of the disease is difficult, but for the clinical aspect of the nidus, its cutaneous surface under the skin was consistent with the levels reached by the BFVols in the afferent arteries. Here, the level of BFVols in the afferent arteries measured once was used to evaluate the activity of AVM qualitatively.

The article "Blood Flow and Shear Stress Allow Monitoring of Progression and Prognosis of Tumor Diseases" was published in 2021. Journal: Front Physiol.

Wall shear stress is a reliable and early biomarker of the progression of abnormal vascular networks. Determination of the WSS in >0.50 cm diameter afferent conduit arteries upstream the pathological local vascular network of PC and AVM shows that for WSS higher than 12.1 dynes/cm^2^ in the SMA or in the ECA: (1) the tumor vascular network continues to expand, (2) the arterial remodeling process is not achieved, and (3) the progression of the disease is then predictable. The delayed achievement of the arterial remodeling in the native artery corresponding to a normalization of the WSS could reflect the stability of PMP or superficial AVM, whatever the level of the BFVol (Figure 1). In AVM, the cutoff for WSS is superior in the smallest native arteries close to the lesion: 25.0 dynes/cm^2^ in afferent arteries of about 0.16 cm inner diameters, i.e., FA or STA. Moreover, the use of WSS seems more accurate and sensitive than the use of BFVol for the prediction of disease progression in all studied arteries.

Patients with complete surgical resection showed similar hemodynamic parameters compared to controls. Resection of the abnormal vascular network decreased the blood flow in the native afferent arteries, resulting in decreased inner diameters. The normalized BFVols with normalized BFVels WSS and inner diameters recorded in those patients were suggestive of a completed ***regressive vascular remodeling***in the afferent arteries as previously demonstrated (Langille and O'Donnell, 1986). Conversely, persistence of high BFVels and high WSSs in the upstream arteries was found in patients with an active progressive disease and was indicative of an ongoing ***expansive vascular*** ***remodeling***.

Arterial remodeling requires coordinated changes in cellular proliferation, apoptosis, migration, cell organization, and matrix-integrin interactions throughout the layered structure of the vessel (Campinho et al., 2020). The association of blood flow with arterial remodeling has been studied in various experimental conditions. In this regard, one of the most comprehensive models to investigate small artery response was developed by Jo de Mey. Persistent changes in blood flow were induced in juvenile rats by ligating every other first-order side branch of the SMA. Thus, patent arteries were exposed to high flow (roughly two times than that normally observed), while occluded mesenteric arteries had practically no blood flow. This chronic low flow resulted in decreased passive lumen diameter, hypotrophy of the artery wall, and both loss and atrophy of smooth muscle cells. On the contrary, high flow led to increased lumen diameter and arterial wall hypertrophy. The completion of the vascular remodeling process required 14–16 days in both low-flow and high-flow arteries, and both conditions are associated with apoptotic cell death (Pourageaud and De Mey, 1998; Buus et al., 2001). In the rabbit, Tronc et al. evidenced the enlargement of the CCA after the creation of an arteriovenous fistula between the CCA and the jugular vein (Tronc et al., 1996).

The article "Blood Flow and Shear Stress Allow Monitoring of Progression and Prognosis of Tumor Diseases" was published in 2021. Journal: Front Physiol.

Lu et al. reported that superficial stage 3 AVMs according to the Schobinger classification showed a higher level of Stromal cell-Derived Factor-1 (SDF-1), Hypoxia-Inducible Factor 1 alpha (HIF-1alpha), and Vascular Endothelial Growth Factor-Receptor (VEGF-R) than stage 2 AVMs. CD133+ and CD34+ endothelial cells were also more frequently expressed in stage 3 AVMs than in stage 2 (Lu et al., 2011). These endothelial progenitor cells are released by the bone marrow in the blood circulation and are responsible for the neovascularization of ischemic lesions or tissues (Rafii and Lyden, 2003). These results suggest that the neoangiogenesis of superficial AVM is at least partially mediated by an ischemic neoangiogenesis mediated by the VEGF. Low-tissue perfusion and consecutive healthy tissues necrosis seem to stimulate the AVM angiogenesis and lead to the development of the AVM. This might explain the paradoxical growth of superficial AVMs after proximal or insufficient embolization, compounding the ischemia of surrounding healthy tissues (Hashimoto et al., 2005; Chen et al., 2008; Buell et al., 2014). Another similar pseudo-pathological state is the artificial arteriovenous (AV) fistula in chronic hemodialysis. It is now known that hemodialysis patients have elevated rates of serum VEGF, soluble intercellular adhesion molecules (sICAM-1), and soluble vascular cell adhesion molecules (sVCAM-1) (Musiał and Zwolińska, 2002; Papayianni et al., 2002; Fadel et al., 2014). Increased levels of VEGF were also demonstrated in patients with occluded AV fistulas compared with patients with nonoccluded AV fistulas (Zohny and Abd el-Fattah, 2008).

In human atherosclerosis, there is ample evidence of active vascular remodeling during the early stages of the disease prior to significant lumen stenosis (Heagerty et al., 1993). The inability of the endothelium to couple the hemodynamic events efficiently to the production of NO has been extensively studied; it contributes to more delayed vascular remodeling in many vascular diseases such as hypertension and diabetes with possible consecutive alteration of the tissues and organs perfusion leading to hypoperfusion and possible ischemia (Rudic and Sessa, 1999).

The article "Blood Flow and Shear Stress Allow Monitoring of Progression and Prognosis of Tumor Diseases" was published in 2021. Journal: Front Physiol.

Oshinski et al. reported spatial-average-time-average WSS of 8.0 ± 4.1 dynes/cm^2^ in the CCA of healthy volunteers (Oshinski et al., 2006). In this study, we found a mean WSS of 10.7 ± 3.3 dynes/cm^2^; the difference may be explained by the different methods of measurement. Indeed, they studied WSS using angio-magnetic-resonance (ARM) imaging. In an older study using Doppler ultrasound, Samijo et al. reported WSS in the CCA of 13 ± 3 dynes/cm^2^ in healthy men and 12 ± 2 dynes/cm^2^ in healthy women. Here, we decided to compute the WSS from ultrasound data in afferent arteries during diseases with highly elevated blood flows. The majority of previous studies exploring the WSS alterations used ARM in ascending or abdominal aorta or carotids during aneurysm or atherosclerotic diseases (Wu et al., 2004, Greve et al., 2006; Efstathopoulos et al., 2008a,b; Peng et al., 2017; Piatti et al., 2017). The purpose of this study was to establish a reliable method of calculation with a noninvasive, affordable, easily accessible exam and, above all, with little or no post-processing tasks. Nevertheless, future users who will measure arterial diameters and BFVels with the Doppler ultrasound method must be aware of the possible variations obtained in the absolute value of the BFVels depending on the ultrasound apparatus they will use, and of course, about the possible shift in the thresholds and cutoffs indicated in this study. They must probably test and recalculate the control values of diameters, BFVels, BFVols, and WSSs given by their ultrasound apparatus and calculate a correction coefficient before using our thresholds and cutoffs directly. Nevertheless, applying the concept of non-achieved or achieved arterial remodeling to differentiate between stable and progressive disease remains true.

Retrospective studies reported that the afferent arteries upstream intracranial AVMs showed elevated WSS before treatment compared to that of the contralateral arteries and that the WSS decreased after treatment (Alaraj et al., 2015). Small vessels diameters and BFVols were also decreased after treatment. Furthermore, Rossiti and Svendsen had previously reported that the inner diameters, the BFVels, and the BFVols were higher in the afferent arteries of intracranial AVMs than in the contralateral side, but there was no difference in the WSS (Rossitti and Svendsen, 1995). They concluded that the arterial remodeling through the increase of the inner diameter was responsible for the normalization of the WSS. In addition, the authors suggest the use of WSS measurement to help determine disease progression with abnormal neoformed vascular network development, such as superficial OPC, PMP, and AVM.

The article "Blood Flow and Shear Stress Allow Monitoring of Progression and Prognosis of Tumor Diseases" was published in 2021. Journal: Front Physiol.

Plasma or tissue tumor markers have been suggested as prognosis factors to monitor treatment response and detect tumor recurrence in gastrointestinal tumors. CEA and CA 19-9 have been mostly investigated. However, treatment decisions should not be based solely on an increased CEA or CA 19-9 (Duffy et al., 2010). In the two preliminary studies with patients with PMP, both tumor markers did not reach the statistically significant level because of the wide distribution of the individual values (Dohan et al., 2017, Barral et al., 2019). Dohan et al. reported that postoperative BFVols after incomplete surgery in patients with PMP might aid in identifying patients who may benefit from postoperative therapy. More precisely, they reported that BFVol was superior in patients with incomplete cytoreductive surgery and active progressive disease than in patients with slow progressive disease. In addition, they found that a cutoff of 530 ml/min could discriminate between slow progressive and active progressive disease with an AUC of 0.827 (95% CI: 0.565–1.00) (*p* < 0.0001). In the present study, similar results were found with a larger number of included patients, and the use of the WSS demonstrated higher performances for discrimination with an AUC = 0.978 (95% CI: 0.902 to 0.999), (*p* < 0.0001).

In conclusion, (1) Doppler ultrasound-derived blood flow calculated in afferent arteries of peritoneal carcinomatosis of the ovarian origin or PMP can easily be used to predict tumor burden, (2) Doppler ultrasound-derived WSS calculated in afferent arteries of PMP or of AVM can easily be used to predict progression. A one-time Doppler ultrasound examination is needed, although progression is usually stated on the modifications showed by modifications between two successive morphological radiological examinations (MDCT and MRI). Although the results of this study are based on specific diseases, the proof of concept could be extrapolated to other diseases with pathological angiogenesis connecting to abnormal vascular networks.

## Data Availability Statement

The raw data supporting the conclusions of this article will be made available by the authors, without undue reservation.

## Ethics Statement

The studies involving human participants were reviewed and approved by Comité de Protection des Personnes Hôpital de Bicêtre 78 rue du général Leclerc 94270 Le Kremlin-Bicêtre. The patients/participants provided their written informed consent to participate in this study.

The article "Blood Flow and Shear Stress Allow Monitoring of Progression and Prognosis of Tumor Diseases" was published in 2021. Journal: Front Physiol.

## Author Contributions

MB, IE-S, and PB performed the Doppler ultrasound acquisitions. All authors participated in the design and writing of the manuscript.

## Conflict of Interest

The authors declare that the research was conducted in the absence of any commercial or financial relationships that could be construed as a potential conflict of interest.

## Publisher's Note

All claims expressed in this article are solely those of the authors and do not necessarily represent those of their affiliated organizations, or those of the publisher, the editors and the reviewers. Any product that may be evaluated in this article, or claim that may be made by its manufacturer, is not guaranteed or endorsed by the publisher.
